# DAFLNet: Dual Asymmetric Feature Learning Network for COVID-19 Disease Diagnosis in X-Rays

**DOI:** 10.1155/2022/3836498

**Published:** 2022-08-09

**Authors:** Jingyao Liu, Jiashi Zhao, Liyuan Zhang, Yu Miao, Wei He, Weili Shi, Yanfang Li, Bai Ji, Ke Zhang, Zhengang Jiang

**Affiliations:** ^1^School of Computer Science and Technology, Changchun University of Science and Technology, Changchun, Jilin 130022, China; ^2^School of Computer and Information Engineering, Chuzhou University, Chuzhou 239000, China; ^3^Zhongshan Institute of Changchun University of Science and Technology, Zhongshan, China; ^4^The First Hospital of Jilin University, Changchun, Jilin, China

## Abstract

COVID-19 has become the largest public health event worldwide since its outbreak, and early detection is a prerequisite for effective treatment. Chest X-ray images have become an important basis for screening and monitoring the disease, and deep learning has shown great potential for this task. Many studies have proposed deep learning methods for automated diagnosis of COVID-19. Although these methods have achieved excellent performance in terms of detection, most have been evaluated using limited datasets and typically use a single deep learning network to extract features. To this end, the dual asymmetric feature learning network (DAFLNet) is proposed, which is divided into two modules, DAFFM and WDFM. DAFFM mainly comprises the backbone networks EfficientNetV2 and DenseNet for feature fusion. WDFM is mainly for weighted decision-level fusion and features a new pretrained network selection algorithm (PNSA) for determination of the optimal weights. Experiments on a large dataset were conducted using two schemes, DAFLNet-1 and DAFLNet-2, and both schemes outperformed eight state-of-the-art classification techniques in terms of classification performance. DAFLNet-1 achieved an average accuracy of up to 98.56% for the triple classification of COVID-19, pneumonia, and healthy images.

## 1. Introduction

COVID-19 is a highly contagious disease originating from severe acute respiratory syndrome coronavirus 2 (SARS-CoV-2). Since its appearance in December 2019, it has spread throughout the globe, which has forced countries to take drastic measures, including closing borders, canceling flights, and quarantining people in countries with related cases. Containing the virus spread appears to be a challenging task [1]. Due to the critical health risks associated with it, COVID-19 was declared by the World Health Organization (WHO) as an international public health emergency and pandemic on 30/01/2020 and 11/03/2020, respectively. As of June 20^th^, 2022, cumulative 524.17 million confirmed COVID-19 cases and 6.34 million deaths worldwide have been reported [2]. Although China has currently contained the epidemic, the situation in some other countries remains dire, and major outbreaks due to SARS-CoV-2 gene mutations are becoming more rapid [3].

As of this writing, the diagnosis of COVID-19 mainly relies on two strategies. The first approach is based on real-time reverse-transcription polymerase chain reaction (PCR), which is an RNA detection method performed on respiratory secretions obtained from the nasopharynx using swabs. The process takes several hours or days and requires a high level of technical proficiency and experience to identify the signs of COVID-19 infection accurately [4]. The second approach is chest X-ray imaging [5]; radiographs of COVID-19 patients show asymmetric peripheral gross glass opacities that are not present in healthy individuals. Manual interpretation by radiologists is easily influenced by fatigue and emotion, etc. Besides, the diagnosis throughput of human experts is not comparable with that of machines, while early symptoms are difficult to spot and may be overlooked by human experts [6]. Therefore, there exists an urgent need to develop a smarter and more accurate algorithm for the automatic detection of diseases such as COVID-19.

Recently, artificial intelligence has shown rapid growth, and researchers have used it to develop novel approaches to disease diagnosis. For example, Kaluri and Reddy [7] performed image feature region segmentation using modified region growing after preprocessing the image. The images were then classified using a genetic algorithm combined with a fuzzy classifier to optimize the selection law. Rajaraman and Antani [8] opted for phased deep learning strategies to train the network and achieved good results for COVID-19 diagnosis. Panwar et al. [9] investigated three datasets using transfer learning and rendered the features in a more interpretable way using the Grad-CAM visualization method. Similarly, Wang et al. [10] analyzed CT images of multiple patients and provided guiding opinions for the diagnosis of the disease. In one work, Rahimzadeh and Attar [11] achieved a classification accuracy of 91.4% using Xception and ResNet50V2 networks for the triple classification of COVID-19, pneumonia, and normal images.

The accuracy of disease diagnosis is mainly influenced by the feature extraction and classification abilities of the network. Related studies from these two aspects are presented next.

First, feature extraction can be improved through feature screening and fusion. Koppu et al. [12] proposed a new method for data cleaning and filtering through the Fitness Oriented Dragonfly Optimization algorithm (F-DA). This method was experimentally proven to be superior to FireFly, gray wolf optimization, and particle swarm optimization for feature filtering. Kaluri and Pradeep Reddy [13] proposed a self-improved genetic algorithm to extract useful features which is more powerful than traditional feature extraction methods. Zhang et al. [14] presented DenseNet with optimized transfer learning and trained the network with comprehensive learning factors, resulting in their proposed DenseNet-OTLS network. The network used optimization of transfer learning setting strategy assigned different learning factors to the frozen, intermediate layer and new layers, and then, training was resumed to find the optimal feature information using some of the parameters learned from migration. Varela-Santos and Melin [15] utilized the gray-level cooccurrence matrix to extract the features through the pooling of two datasets and used a neural network for triple classification, resulting in an accuracy of 98.8%. Moreover, Ozturk et al. [16] utilized a network based on 17 convolutional layers, where each layer used a different filter to extract different features from the different layers. The model was labeled as DarkNet and achieved 98.08% accuracy in dichotomous classification and 87.02% accuracy in multiclassification. All the above algorithms employed single features and did not perform feature fusion. However, multifeature fusion results in a more representation of information and consequently in increased accuracy. For instance, Chen et al. [17] used ResNet and DenseNet to extract features and weighted them with multiple classifiers to classify 14 lung diseases (the model is called DualCheXNet). Likewise, Wang et al. [18] collected images from local hospitals and used an improved transfer learning method to introduce two networks, DenseNet and ResNet, for discriminant correlation analysis feature fusion and further classification (CCSHNet model). Recently, Wang et al. [6] utilized the GCN as a backbone network and proposed a deep feature fusion method with high classification accuracy for COVID-19.

Second, the network's classification capability can be improved through the replacement of classifiers or by performing decision-level fusion. For example, similarly, Toğaçar et al. [19] trained deep learning models (MobileNetV2 and SqueezeNet) on three datasets and used an SVM as a classifier for data classification, thus not only utilizing a deep learning network framework but also applying machine learning methods. Chen et al. [17] improved classification accuracy by balancing three classifiers for decision-level fusion for the identification of fourteen lung diseases and provided experimental evidence of their method's effectiveness. Canayaz [20] used SVM to replace the original deep learning fully connected layer in order to improve the classification accuracy after feature filtering using two metaheuristic algorithms, resulting in 99.38% accuracy for COVID-19 multiclassification.

In past studies, the use of separate networks to extract features was common but did not result in the extraction of rich features. Furthermore, most methods used one classifier with an unbalanced classification ability, which led to a low diagnostic performance. In this paper, both feature extraction capability and disease classification capability are taken into account through the use of two separate networks to extract features for fusion. In this manner, the feature extraction capability is improved. Then, the weighted decision results of three classifiers are used to improve classification capability. Disease feature learning and disease diagnosis results are influenced by the size of the dataset, and many past studies have commonly used datasets with a small number of images. In contrast, in this study, a dataset with 9208 images with rich samples is used. Also, a spatial attention mechanism module and a channel attention mechanism module are introduced in the network to further improve its feature extraction ability.

From the technical point of view, the main contributions of this work are as follows:

1. The efficient classification model DAFLNet is proposed, which consists of two modules, the dual asymmetric feature-level fusion module (DAFFM) and the weighted decision-level fusion module (WDFM). In addition, two schemes are proposed, which are DAFFM-1 and DAFFM-2
2. The proposed model employs both pixel-level fusion and weighted decision-level fusion
3. To determine the optimal weights for weighted decision-level fusion, a new pretrained network selection algorithm (PNSA) is proposed
4. Multiway data augmentation is performed on chest X-ray images (CXRs) to improve sample diversity
5. Compared to 8 state-of-the-art diagnosis methods for COVID-19, experimental results show that DAFLNet is effective and gives better performance

The structure of this paper is organized as follows. An overview of recent attempts to detect COVID-19 in medical images and the relevant studies reported in this regard are first presented. In Section 2, the dataset, the involved deep learning methods, and the proposed new model are described. Subsequently, in Section 3, the data preprocessing methods are presented along with the experimental steps and methods. The experimental results are also discussed, analyzed, and compared with the existing methods. Finally, in Section 4, a summary of the paper is presented.

## 2. Dataset and Methods

This section comprises four parts. First, the dataset and preprocessing methods are introduced. The second part describes the deep learning networks, while the third part introduces the two modules proposed in this paper. Finally, the proposed method is described in detail.

### 2.1. Dataset

#### 2.1.1. Original Dataset

Sait et al. [21] collected 15 publicly available COVID-19 datasets and removed the duplicates to form a new dataset, which is the one used in this work. The dataset contains 1281 COVID-19 X-rays, 1656 viral pneumonia X-rays, 3270 normal X-rays, and 3001 bacterial pneumonia X-rays. The viral pneumonia and bacterial pneumonia were combined in a single category. The dataset included images from both children and adults. Three randomly selected images from the three categories are shown in Figure 1.

#### 2.1.2. Dataset Preprocessing

The dataset contained healthy, COVID-19, and pneumonia X-ray images, marked as H, C, and P, as expressed in Equation (1). If the input image size is large, it is likely that redundant information present will slow down the processing speed of the neural network, so the set *X* of original images was resized to a uniform size of 224 × 224, and a new image set *Y* was obtained, as shown in Equation (2):

(1) $$\begin{array}{c} X=\left\{H,C,P\right\}, \end{array}$$

(2) $$\begin{array}{c} Y=\text{Resize}\left(X,\left[224,224\right]\right)=\left\{x_{1},x_{2},x_{3}\cdots ,x_{n}\right\}. \end{array}$$

The size reduction also improved the overall storage memory requirements substantially. Intuitively, it can be observed that this resizing operation can decrease the storage size required by 1 − (224 × 224 × 3 × 4)/(1024 × 1024 × 3 × 4) = 95.21%, thus enabling the storage of all CXRs in RAM, which accelerates the speed for the proposed algorithms.

In our experiments, the dataset was randomly divided into three subsets: the training set (*A*: 70%), the validation set (*B*: 10%), and the test set (*C*: 20%). The relevant information is listed in Table 1.

### 2.2. Deep Learning Models

#### 2.2.1. EfficientNetV2

EfficientNet [22] is a balance input image size, network depth, and width to obtain the best results. In this study, EfficientNetV2 [23] was used as the backbone network. Fused-MBConv is the core part of EfficentNetV2 and replaces the 1 × 1 boosting convolution and 3 × 3 depth-wise convolution operations of MBConv with normal 3 × 3 convolution to reduce training times. EfficentNetV2 is approximately ten times faster than EfficientNet in training and has better performance [24].  Figure 2 illustrates the structure of MBConv and Fused-MBConv. In addition, with EfficientNetV2, the whole training process is divided into four stages, and a progressive learning strategy with strong regularization is used in each stage, resulting in a network with few parameters and high accuracy.

#### 2.2.2. DenseNet+CBAM

DenseNet (Dense Convolutional Network) was proposed by Huang et al. [25]. It connects each layer with other layers in a feed-forward fashion. In traditional convolutional neural networks, the network has *L* connections for *L* layers, while in DenseNet, there are *L* · (*L* + 1)/2 connections, and the input of each layer comes from the output of all the previous layers. DenseNet consists of DenseBlock and a transition layer. In DenseBlock, the size of each layer does not change, and the channel dimension changes. Suppose the output of each nonlinear transformation *H* is *K* feature maps. Then, the input of the network in layer *i* will be *K*_0_ + (*i* − 1) × *K*. The structure of DenseNet is shown in Figure 3. DenseNet121 and DenseNet169 were used for this study's experiments.

The convolutional block attention module (CBAM) [26] is separated into two distinct parts, referred to as the channel attention (CA) module and the spatial attention (SA) module. This not only results in a reduced number of parameters and computational cost but also allows its integration as a plug-and-play module to existing network architectures. Each channel of a feature represents a specialized detector; therefore, channel attention is focused on features that are meaningful. To aggregate spatial features, CBAM uses both global average and maximum pooling to exploit different aspects of the information, separately. Besides, CBAM introduces a spatial attention module to concentrate on meaningful features. Since EfficientNetV2 has an integrated SE attention module, in this paper, we add CBAM to DenseNet so that both networks can utilize useful information and achieve good feature extraction capability. Then, the outputs of the two networks are fused to enrich the extracted features' characteristics.

### 2.3. Feature-Level Fusion Module

EfficientNetV2 and DenseNet acquire features in different ways, and they are fused to acquire different features. In DAFFM, these two deep learning networks extract features in parallel. Two schemes are proposed, called DAFLNet-1 and DAFLNet-2, where DAFLNet-1 consists of EfficientNetV2 and DenseNet121, while DAFLNet-2 consists of EfficientNetV2 and DenseNet169.

The information fusion is divided into three levels: pixel-level fusion (PLF), feature-level fusion (FLF), and decision-level fusion (DLF). Commonly, there exist two feature fusion methods concat and add. Add corresponds to an increase in information amount for the features describing the image; however, the dimensions describing the image do not increase; only the amount of information under each dimension is increasing. On the other hand, concat refers to a merger of the number of channels, i.e., the number of channels describing the image increases, while relevant information for each feature stays constant. The relevant mathematical expressions are given in Equations (3) and (4). In this study, we used concat for feature-level fusion, as shown in Figure 4. The number of Fusion_Feature1_Feature2 channels refers to the sum of Feature1 and Feature2 channels:

(3) $$\begin{array}{c} F_{flf}=\text{concat}\left(F_{E},F_{D}\right), \end{array}$$

(4) $$\begin{array}{c} F_{flf}=\text{add}\left(F_{E},F_{D}\right), \end{array}$$

where *F*_*E*_ is the feature extracted by EfficientNetV2, *F*_*D*_ is the feature extracted by DenseNet, and *F*_*flf*_ is the fused features' set.

### 2.4. Pretrained Network Selection Algorithm

There are three types of features in WDFM. The first one is extracted by EfficientNetV2, the second one is extracted by DenseNet, and the third one is obtained through the fusion of the two network outputs, which are both related and different. The three types correspond to three classifiers, auxiliary classifier1, auxiliary classifier2, and the fusion classifier. Experiments have shown that one classifier is not effective and that three classifiers with different weights can achieve better results. Thus, the loss of DAFLNet is

(5) $$\begin{array}{c} L=w_{E}L_{E}+w_{D}L_{D}+w_{F}L_{F}, \end{array}$$

where *L*_*E*_, *L*_*D*_, and *L*_*F*_ are the losses corresponding to the three classifiers, while *w*_*E*_, *w*_*D*_, and *w*_*F*_ are the weights corresponding to the three losses. Since different features enable different classification capabilities for the results, the greedy selection algorithm is unsuitable for the determination of weights because it does not guarantee that the fusion-based classification will yield the best performance. Therefore, a new pretrained network selection algorithm (PNSA) is proposed, which will aid the selection of the optimal weights in the range. The pseudocode of PNSA is presented in Algorithm 1. In this study, the fusion features are considered to be the richest, so *w*_*F*_ is set to 1. The two auxiliary classifiers serve the same purpose, so *w*_*E*_ = *w*_*D*_. The system's performance was analyzed for different values of *w*_*E*_ and *w*_*D*_, denoted as Concat0 (*w*_*F*_ = 1.0, *w*_*D*_ = *w*_*R*_ = 0), Concat1 (*w*_*F*_ = 1.0, *w*_*D*_ = *w*_*R*_ = 0.1), Concat2 (*w*_*F*_ = 1.0, *w*_*D*_ = *w*_*R*_ = 0.2), Concat3 (*w*_*F*_ = 1.0, *w*_*D*_ = *w*_*R*_ = 0.3), Concat4 (*w*_*F*_ = 1.0, *w*_*D*_ = *w*_*R*_ = 0.4), and Concat5 (*w*_*F*_ = 1.0, *w*_*D*_ = *w*_*R*_ = 0.5). We finally determined that the network performance was best when *w*_*F*_ was set to 1 and *w*_*E*_ and *w*_*D*_ were set to 0.4.

### 2.5. Proposed Approach

DAFLNet is mainly used for disease classification of chest X-ray images where COVID-19 has caused the appearance of ground glass-like shadows. In order to obtain richer features from limited images, four approaches for multiple-way data augmentation were adopted. The proposed approach is divided into two modules: DAFFM and WDFM, which improve the network performance in terms of both feature extraction and classification ability, respectively. DAFFM uses the EfficientNetV2 and DenseNet deep learning models, with CBAM added to DenseNet, and the features extracted by the two networks are fused to improve the feature extraction capability. The weighted classification fusion strategy is used in WDFM to improve the disease prediction accuracy.  Figure 5 shows the overall design of the proposed method. To elaborate further, a pseudocode for DAFLNet is given in Algorithm 2.

## 3. Experimental Analysis and Results

### 3.1. Experiment Platform

In this experiment, Python language was used for implementation and data preprocessing. The hardware utilized was a 32 GB Tesla V100 graphics card and an Intel® Xeon® CPU E5-2698 v4 @ 2.20 GHz processor running the Linux operating system. Libraries such as numpy and the deep learning pytorch toolbox were used. The learning rate (LR), batch size (BS), epochs, optimizer, and dropout rate (DR) made up the tuned hyperparameters of the model. The values listed in Table 2 produced the optimal experimental results. When the loss diminished, the LR was decreased to its original value of 0.1. The training process was terminated when the training loss threshold exceeded 3 times and the value obtained was not less than that of the previous iteration.

### 3.2. Data Augmentation

To mitigate any potential overfitting, multiway data augmentation (MDA) [6] was utilized. As shown in Figure 6, we used four ways to enhance the training data (*A*). Furthermore, through the random hold-out (RHO) method, the resized dataset *Y* was partitioned into three sections: the training set *A*, the validation set *B*, and the test set *C*:

(6) $$\begin{array}{c} Y\overset{\text{RHO}}{⟶}\left\{A,B,C\right\}, \end{array}$$

where

(7) $$\begin{array}{c} A=\left\{a\left(i\right)\right\},\\ B=\left\{b\left(i\right)\right\},\\ C=\left\{c\left(i\right)\right\}, \end{array}$$

and the relevant sizes related to these subsets satisfy the following equation:

(8) $$\begin{array}{c} \left|Y\right|=\left|A\right|+\left|B\right|+\left|C\right|, \end{array}$$

where ∣·∣ refers to the cardinality of a set.

Assuming that there are *k*_MDC_ MDA techniques, and *n*_MDA_ images are generated using each technique; eventually, *k*_MDC_ × *n*_MDA_ images are generated. The following four MDA methods were used in this study.

#### 3.2.1. Noise Injection (N_I)

Gaussian noise was injected into all the images of a training set, thereby generating new noisy images:

(9) $$\begin{array}{c} \left.\overset{⟶}{z^{A1}\left(i\right)}\right|=F_{\text{N}\_\text{I}}\left[z^{A}\left(i\right)\right]=\left[z^{A1}\left(i\right),\cdots ,z_{n_{\text{MDA}}}^{A1}\left(i\right)\right], \end{array}$$

where *F*_N_I_ denotes the noise injection function.

#### 3.2.2. Rotation (Ro)

The rotation angle *θ*^Ro^ = 90° was applied to the images:

(10) $$\begin{array}{c} \left.\overset{⟶}{z^{A2}\left(i\right)}\right|=F_{\text{Ro}}\left[z\left(i\right)\right]=\left[z^{A2}\left(i,\theta_{1}^{\text{Ro}}\right),\cdots ,z_{n_{\text{MDA}}}^{A2}\left(i,\theta_{n_{\text{MDA}}}^{\text{Ro}}\right)\right], \end{array}$$

where *F*_Ro_ corresponds to the function of rotation.

#### 3.2.3. Gamma Correction (G_C)

The gamma correction factor r^G_C^ =1.5 was used to produce new images as follows:

(11) $$\begin{array}{c} \left.\overset{⟶}{z^{A3}\left(i\right)}\right|=F_{\text{G}\_\text{C}}\left[z\left(i\right)\right]=\left[z^{A3}\left(i,r_{1}^{\text{G}\_\text{C}}\right),\cdots ,z_{n_{\text{MDA}}}^{A3}\left(i,r_{n_{\text{MDA}}}^{\text{G}\_\text{C}}\right)\right], \end{array}$$

where *F*_G_C_ refers to the gamma correction function.

#### 3.2.4. Mirror (Mir)

(12) $$\begin{array}{c} \left.\overset{⟶}{z^{A4}\left(i\right)}\right|=F_{\text{Mir}}\left[z\left(i\right)\right]=\left[z^{A4}\left(i\right),\cdots ,z_{n_{\text{MDA}}}^{A4}\left(i\right)\right], \end{array}$$

where *F*_Mir_ is the mirroring function.

### 3.3. Evaluation Metrics

To assess the performance of the proposed DAFLNet method, various indicators were concurrent, namely, accuracy (Acc), precision (Pre), sensitivity (Sen), specificity (Spe), recall (Rec), and F1-score (F1‐sc). The true positives (TP), true negatives (TN), false positives (FP), and false negatives (FN) were used to identify the diagnosis of CXRs by the model. A TP indicates a positive outcome for both the real category of the sample and the recognition result. Similarly, a FN highlights a positive real category of the sample identified as negative by the model. Alternatively, FP refers to a negative real category of the sample recognized as a positive by the model. Finally, a TN indicates a negative real sample category recognized as such correctly. The corresponding equations are expressed below:

(13) $$\begin{array}{c} \text{Acc}=\frac{\text{TP}+\text{TN}}{\text{TP}+\text{TN}+\text{FP}+\text{PN}},\\ \text{Pre}=\frac{\text{TP}}{\text{TP}+\text{FP}},\\ \text{Sen}=\frac{\text{TP}}{\text{TP}+\text{FN}},\\ \text{Spe}=\frac{\text{TN}}{\text{TN}+\text{FP}},\\ \text{Rec}=\frac{\text{TP}}{\text{TP}+\text{TN}},\\ \text{F}1‐\text{sc}=\frac{2*\text{Pre}*\text{Rec}}{\text{Pre}+\text{Rec}}. \end{array}$$

### 3.4. Feature-Fusion Methods and Decision-Level Fusion Weight

In our experiments, a comparative study was performed to determine the fusion method. Both concat and add fusion were performed for DAFLNet-1 and DAFLNet-2, and the corresponding results from the experiment are given in Figure 7. Generally, the concat results yielded better performance compared to add, so the concat method was chosen for the ensuing experiments.

The weight of decision-level fusion determines the performance of the network. Experiments were conducted using DAFLNet-1 and DAFLNet-2 to determine the optimal values of *w*_*E*_, *w*_*D*_, and *w*_*F*_ experimentally. The results are shown in Figure 8. The best performance is achieved when *w*_*F*_ = 1 and *w*_*E*_ = *w*_*D*_ = 0.4, with DAFLNet-2 exhibiting better performance than DAFLNet-1.

### 3.5. Proposed DAFLNet

In order to determine the optimal fusion strategy, the two schemes DAFLNet-1 and DAFLNet-2 were tested under different configurations. This process comprised a total of 9 stages M1, ⋯, M9, as shown in Table 3.

### 3.6. Experimental Results

#### 3.6.1. Effect of DAFLNet

The experiment was conducted five times, and the best results in the test set are shown in Table 4. M4 and M5 were more accurate than M1, M2, and M3, thus highlighting that the fused networks were generally more effective than the individual networks. Besides, M6 and M7 were based on M4 and M5 through the addition of the convolutional block attention module (CBAM) to ResBlock. The experimental results show that the performance of the networks with the addition of CBAM was improved.  Figure 9 illustrates the overall performance of the nine networks visually. Finally, the performance of the network was further improved through the addition of weighted decision-level fusion, where DAFLNet-1 achieved a classification accuracy of 98.86%.

#### 3.6.2. Classification Performance Validation

To illustrate the classification of data from the validation set of 921 CXRs, a confusion matrix [27] was created. Figures 10 and 11 show the confusion matrix of the proposed DAFLNet-1 and DAFLNet-2 models.

Table 5 demonstrates the overall performance of DAFLNet-1 and DAFLNet-2 for the validation set, revealing an average accuracy of 99.61%, 98.63%, and 98.41% for COVID-19, pneumonia, and normal X-ray images for DAFLNet-1, respectively. The average accuracy in DAFLNet-2 was 99.56%, 98.52%, and 98.31% for COVID-19, pneumonia, and normal X-ray images, respectively. In conclusion, the DAFLNet proposed in this paper performed well in terms of accuracy, recall, and F1-score even with unbalanced data.

#### 3.6.3. Comparison with State-of-the-Art Approaches

To demonstrate the proposed method's contribution, the proposed DAFLNet method was compared with 8 state-of-the-art approaches: ECOVNet-EfficientNetB3 base [28], BCNN_SVM [29], COVNet [30], DTL-V19 [9], DenseNet121 [31], Resnet50V2 [32], Xception [33], and MobileNetV2 [34]. The same dataset with all methods and the results shown are the mean and standard deviation of 5 runs.  Table 6 illustrates the relevant comparison results.

Compared to the other methods, the strategy proposed in this work is unique. BCNN_SVM used a BCNN bilinear fusion of two deep learning networks, VGG16 and VGG19, to extract the features, and then used an SVM to classify for the presence of COVID-19. Since both fusion networks were based on VGG, the extracted features were similar and the relevant accuracy was lower than the proposed DAFLNet. Additionally, the DTL-V19 of the work in question used deep migration learning to migrate VGG19 over to COVID-19 classification. This resulted in fewer training parameters; nevertheless, the network layers were fewer, resulting in limited performance and overfitting. ECOVNet-EfficientNetB3 and COVNet use EfficientNetB3 and ResNet50, respectively, as pretrained networks for classification. These are models, so their performance is inferior compared to the proposed network owing to the absence of feature fusion. Furthermore, the proposed method was compared with the currently popular classification networks, namely, DenseNet121, Resnet50V2, Xception, and MobileNetV2, and results indicate that these networks are not as effective as DAFLNet.

DAFLNet takes into account both feature extraction and disease classification, using two networks to extract features for fusion, thus resulting in improved feature extraction capability, while the weighted classification results of the three classifiers improve its classification capability. It can be seen that, among all methods, the proposed DAFLNet achieved the best results. Moreover, DAFLNet-1 achieved an average accuracy of 98.56%, and DAFLNet-2 achieved an average accuracy of 98.41%. The high accuracy was mainly achieved through the coordinated feature fusion and attention mechanisms, the use of the newly proposed EfficientNetV2 as the backbone network, and the utilization of an improved classifier, the effectiveness of which is demonstrated through the experimental results. In addition, the proposed multiplexed data augmentation prevents model overfitting, hence improving its performance.

## 4. Conclusions

In this paper, the Chest Lesion Feature Fusion Network (DAFLNet) is proposed, which achieved an average accuracy of 98.56%. From the performance perspective, the network can diagnose COVID-19, health, and pneumonia accurately. To validate the performance of DAFLNet, it was compared to 8 state-of-the-art methods on two datasets. The experimental results showed that DAFLNet achieved the best detection performance in terms of accuracy, precision, sensitivity, and F1-score on both datasets. From the perspective of computational efficiency, DAFLNet fusion with two deep learning networks and CBAM results in longer training times, which is a disadvantage. However, the model obtained after training can diagnose the disease quickly and has similar diagnostic speed to the other methods. In terms of generalization ability, the proposed method can extract more disease features for diagnosis. With regard to practicality, DAFLNet can be deployed to hospital servers to assist doctors in faster and more accurate diagnosis, making a significant contribution to society and hospitals.

The comparison of this method with other methods illustrates its effectiveness. However, the method has not been validated on CT images. Furthermore, the proposed method utilizes a large number of parameters due to the fusion of two networks performed. Thus, future research directions will be towards the reduction of the number of parameters and experimentation on different types of datasets.

## Figures and Tables

**Figure 1:** Sample images of the (a) COVID-19, (b) normal, and (c) pneumonia chest category X-rays.

**Figure 2:** Structure of MBConv and Fused-MBConv.

**Figure 3:** DenseNet structure.

**Figure 4:** Concat for feature-level fusion.

**Figure 5:** Structure of the proposed DAFLNet.

**Figure 6:** Samples from the original and the enhanced dataset.

**Figure 7:** Comparison experiment of the concat and add methods.

**Figure 8:** Average accuracy scores of DAFLNet-1 and DAFLNet-2 with different decision-level fusion weights.

**Figure 9:** Optimal performance results of the nine networks.

**Figure 10:** Classification results of DAFLNet-1 visualized using a confusion matrix.

**Figure 11:** Classification results of DAFLNet-2 visualized using a confusion matrix.

**Algorithm 1:** Proposed PNSA for weight selection.

**Algorithm 2:** Pseudocode of DAFLNet algorithm.

**Table 1:** Data distribution in the model.

Dataset	Test (20%)	Training (70%)	Validation (10%)	Total
COVID-19	256	897	128	1281
Normal	654	2289	327	3270
Pneumonia	931	3260	466	4657
Total	1841	6446	921	9208

**Table 2:** Hyperparameters of the DAFLNet network model.

Hyperparameter	Value
LR	0.0003
BS	16
Epochs	30
Optimizer	Adam
DR	0.4

**Table 3:** Nine proposed networks.

Index	Modules	Network name	Description
M1		EfficientNetV2	Backbone network
M2		DenseNet121	Auxiliary network1
M3		DenseNet169	Auxiliary network2
M4	⟵FLF(M1, M2)	Eff-V2&D-121	FLF of M1 and M2
M5	⟵FLF(M1, M3)	Eff-V2&D-169	FLF of M1 and M3
M6	⟵M4 + CBAM	DAFFM-1	Add CBAM to M4
M7	⟵M5 + CBAM	DAFFM-2	Add CBAM to M5
M8	⟵DLF(M1, M2, M6)	DAFLNet-1	DLF of M1, M2, and M6
M9	⟵DLF(M1, M2, M7)	DAFLNet-1	DLF of M1, M2, and M7

**Table 4:** Best accuracy of nine networks in the test set (%).

ID	Model	COVID-19	Normal	Pneumonia	Overall Acc.
M1	EfficientNetV2	98.4	97.50	97.56	97.23
M2	DenseNet121	98.08	97.45	97.18	96.85
M3	DenseNet169	97.91	97.12	97.12	96.58
M4	Eff-V2&D-121	98.35	97.94	98.15	97.61
M5	Eff-V2&D-169	99.13	97.77	97.77	97.34
M6	DAFFM-1	99.13	98.05	98.05	97.72
M7	DAFFM-2	99.51	98.53	98.48	98.26
M8	DAFLNet-1	99.62	99.08	99.02	98.86
M9	DAFLNet-2	99.62	99.13	98.86	98.81

**Table 5:** Classification of DAFLNet networks after two kinds of validation (%).

Models	Class	Acc (c)	Sen (c)	Pre (c)	Rec (c)	Spe (c)	F1-sc (c)	Overall Acc
DAFLNet-1	COVID-19	99.61 ± 0.24	98.44 ± 1.35	98.75 ± 1.02	98.44 ± 1.35	99.80 ± 0.17	98.59 ± 0.86	98.33 ± 0.52
	Normal	98.63 ± 0.39	97.55 ± 0.78	98.58 ± 0.47	97.55 ± 0.78	99.23 ± 0.26	98.06 ± 0.55	
	Pneumonia	98.41 ± 0.43	98.84 ± 0.33	98.04 ± 0.56	98.84 ± 0.33	97.98 ± 0.59	98.44 ± 0.42	
DAFLNet-2	COVID-19	99.56 ± 0.23	98.44 ± 0.55	98.45 ± 1.43	98.44 ± 0.55	99.75 ± 0.24	98.44 ± 0.82	98.20 ± 0.55
	Normal	98.52 ± 0.35	97.06 ± 0.88	98.76 ± 0.44	97.06 ± 0.89	99.33 ± 0.24	97.90 ± 0.50	
	Pneumonia	98.31 ± 0.54	98.93 ± 0.64	97.75 ± 0.61	98.93 ± 0.64	97.67 ± 0.63	98.34 ± 0.53	

**Table 6:** Performance comparison of the proposed DAFLNet with other studies (%).

Method	Class	Sen (c)	Pre (c)	F1-sc (c)	Overall Acc
ECOVNet-EfficientNetB3 base [28]	COVID-19	95.70 ± 1.95	96.77 ± 1.68	96.23 ± 1.6	96.67 ± 0.67
	Normal	96.58 ± 0.7	96.20 ± 0.81	96.38 ± 0.66	
	Pneumonia	97.02 ± 0.80	97.00 ± 0.41	97.01 ± 0.58	
BCNN_SVM [29]	COVID-19	97.58 ± 2.07	98.75 ± 0.88	98.15 ± 0.71	97.76 ± 0.42
	Normal	96.82 ± 0.98	97.85 ± 1.01	97.33 ± 0.54	
	Pneumonia	98.48 ± 0.85	97.46 ± 0.81	97.96 ± 0.40	
COVNet [30]	COVID-19	86.95 ± 3.64	92.19 ± 3.02	89.46 ± 2.68	93.14 ± 1.11
	Normal	92.21 ± 2.24	92.65 ± 1.06	92.38 ± 1.06	
	Pneumonia	95.94 ± 1.34	93.38 ± 0.85	94.64 ± 0.88	
DTL-V19 [10]	COVID-19	92.73 ± 1.86	91.99 ± 3.23	92.35 ± 2.52	91.53 ± 2.14
	Normal	85.44 ± 4.09	92.73 ± 1.44	88.92 ± 2.78	
	Pneumonia	95.47 ± 1.01	90.70 ± 2.51	93.02 ± 1.76	
DenseNet121 [31]	COVID-19	82.97 ± 5.10	90.25 ± 3.87	86.45 ± 4.53	91.99 ± 1.95
	Normal	90.83 ± 20.2	91.44 ± 2.72	91.13 ± 2.21	
	Pneumonia	95.28 ± 1.29	92.80 ± 1.47	94.02 ± 1.24	
Resnet50V2 [32]	COVID-19	87.27 ± 3.80	93.32 ± 2.21	90.17 ± 2.73	93.21 ± 1.19
	Normal	91.25 ± 1.55	93.64 ± 1.42	92.43 ± 1.30	
	Pneumonia	96.22 ± 1.01	92.91 ± 1.20	94.54 ± 0.94	
Xception [33]	COVID-19	94.61 ± 1.31	95.65 ± 2.64	95.10 ± 1.30	94.99 ± 1.02
	Normal	92.97 ± 2.03	94.65 ± 1.47	93.79 ± 1.46	
	Pneumonia	96.52 ± 0.91	95.08 ± 0.85	95.79 ± 0.79	
MobileNetV2 [34]	COVID-19	81.09 ± 6.16	91.01 ± 3.80	85.72 ± 4.84	90.60 ± 2.01
	Normal	90.67 ± 1.50	88.54 ± 3.07	89.58 ± 2.11	
	Pneumonia	93.15 ± 1.54	91.98 ± 1.03	92.56 ± 1.25	
DAFLNet-1 (this work)	COVID-19	97.74 ± 0.43	99.37 ± 0.21	98.54 ± 0.11	98.56 ± 0.39
	Normal	98.13 ± 1.09	98.47 ± 0.21	98.29 ± 0.53	
	Pneumonia	99.10 ± 0.14	98.43 ± 0.83	98.76 ± 0.36	
DAFLNet-2 (this work)	COVID-19	97.97 ± 0.89	99.45 ± 0.35	98.70 ± 0.44	98.41 ± 0.27
	Normal	97.55 ± 0.66	98.82 ± 0.26	98.18 ± 0.35	
	Pneumonia	99.14 ± 0.15	97.86 ± 0.53	98.50 ± 0.24	

## Data Availability

The data that support the findings of this study are open at https://data.mendeley.com/datasets/9xkhgts2s6/1.
